The article "Optimal Facial Feature Based Emotional Recognition Using Deep Learning Algorithm" was published in 2022. Journal: Comput Intell Neurosci.

# Optimal Facial Feature Based Emotional Recognition Using Deep Learning Algorithm

**DOI:** 10.1155/2022/8379202

**Published:** 2022-09-20

**Authors:** Tarun Kumar Arora, Pavan Kumar Chaubey, Manju Shree Raman, Bhupendra Kumar, Yagnam Nagesh, P. K. Anjani, Hamed M. S. Ahmed, Arshad Hashmi, S. Balamuralitharan, Baru Debtera

**Affiliations:** ^1^Professor-Department of Applied Sciences and Humanities, ABES Engineering College, Ghaziabad, Uttar Pradesh, India; ^2^Department of Applied Sciences Engineering, Tula's Institute, Dhoolkot, Dehradun, Uttarakhand, India; ^3^Department of Management College of Business & Economics, Debre Tabor University, Debra Tabor, Ethiopia; ^4^College of Business & Economics, Debre Tabor University Ethiopia, Debra Tabor, Ethiopia; ^5^IT Department, Debra Tabore University, Debra Tabor, Ethiopia; ^6^Department of Management Studies, Sona College of Technology, Salem, TN, India; ^7^Department of Management, College of Business and Economics, Werabe University, Addis Ababa, Ethiopia; ^8^Information Systems Department Faculty of Computing and Information Technology In Rabigh (Fcitr), King Abdulaziz University, Jeddah, Saudi Arabia; ^9^Department of Mathematics, Bharath Institute of Higher Education and Research, Bharath Institute of Science and Technology, No. 173 Agharam Road Selaiyur, Chennai 600 073, Tamil Nadu, India; ^10^Department of Chemical Engineering, College of Biological and Chemical Engineering, Addis Ababa Science and Technology University, Addis Ababa, Ethiopia

## Abstract

Humans have traditionally found it simple to identify emotions from facial expressions, but it is far more difficult for a computer system to do the same. The social signal processing subfield of emotion recognition from facial expression is used in a wide range of contexts, particularly for human-computer interaction. Automatic emotion recognition has been the subject of numerous studies, most of which use a machine learning methodology. The recognition of simple emotions like anger, happiness, contempt, fear, sadness, and surprise, however, continues to be a difficult topic in computer vision. Deep learning has recently drawn increased attention as a solution to a variety of practical issues, including emotion recognition. In this study, we improved the convolutional neural network technique to identify 7 fundamental emotions and evaluated several preprocessing techniques to demonstrate how they affected the CNN performance. This research focuses on improving facial features and expressions based on emotional recognition. By identifying or recognising facial expressions that elicit human responses, it is possible for computers to make more accurate predictions about a person's mental state and to provide more tailored responses. As a result, we examine how a deep learning technique that employs a convolutional neural network might improve the detection of emotions based on facial features (CNN). Multiple facial expressions are included in our dataset, which consists of about 32,298 photos for testing and training. The preprocessing system aids in removing noise from the input image, and the pretraining phase aids in revealing face detection after noise removal, including feature extraction. As a result, the existing paper generates the classification of multiple facial reactions like the seven emotions of the facial acting coding system (FACS) without using the optimization technique, but our proposed paper reveals the same seven emotions of the facial acting coding system.

The article "Optimal Facial Feature Based Emotional Recognition Using Deep Learning Algorithm" was published in 2022. Journal: Comput Intell Neurosci.

## 1. Introduction

Emotional recognition is one of the most crucial and challenging techniques nowadays. Emotion recognition is used in a wide range of applications, like helping to evaluate blood pressure, stress levels, etc. The facial features using emotional techniques include the functions of the application of happy, sad, calm, and neutral. Many of the techniques and algorithms help to detect the interior workings of the human body.

Emotional recognition detects the human being's thoughts at an instant level. It prevents human beings from major infections or diseases just because of the early detection of diseases using emotional recognition. The main advantage of emotional recognition is that it helps to identify human mentalities without asking them.

Much facial recognition is involved in the video-based identification of the various types of emotions without knowing their knowledge. This paper provides two strategies to calculate the video-based face recognition method, namely, the one that is measured with the accuracy of the distance and the angles. And the other one is the arrangement of the all-video clips, which reduces the set of key frames [1].

A wide range of fields, including clinical psychology, psychiatry, neurology, pain assessment, lie detection, intelligent settings, and multimodal human-computer interface, can benefit from the use of automatic facial expressions. Facial expression analysis uses two methods: feature extraction and action unit identification from the facial action coding system (FACS). Ekman et al. suggested the framework known as FACS. Geometric feature-based and appearance-based feature extraction are the two basic methods. In order to create feature vectors and depict the face from a geometrical perspective, the former represents facial points. The latter is used in the extraction of feature vectors, either in a focused or all-encompassing facial image, such as in the use of Gabor Wavelets. Deep learning is a component of machine learning techniques that can be used for facial expression analysis and emotion recognition. However, the amount of data affects how well it performs. The performance improves as the data volume increases. Facial expression dataset sizes are still too small for deep learning to be applied. To enhance the variance and, subsequently, the amount of the data, several studies use augmentation techniques during the preprocessing stage, such as cropping, scaling, translating, or mirroring. These preprocessing methods are very good at enhancing the capabilities of deep learning. This study attempts to demonstrate the effects of data preprocessing on deep learning performance while also employing deep learning to recognise emotions. We evaluate each preprocessing method's accuracy in comparison to the sum of its parts before looking at the accuracy variability.

The article "Optimal Facial Feature Based Emotional Recognition Using Deep Learning Algorithm" was published in 2022. Journal: Comput Intell Neurosci.

The data augmentation algorithm in deep learning techniques helps to reduce the dimensional space of this picture with the help of expanding the training set in the data collection based on the image augmentation technique [2]. This paper implements kernel filters to reduce the sharp edges in the image.

Facial emotions like sadness and stress are accurately calculated by machine learning algorithms. The ECG and the PPG worked with the 28 features extracted in machine learning algorithms to provide better accuracy in the results for the identification of sad and angry like negative emotions [3].

Facial expressions play a crucial role in the identification of human mentality without sharing their knowledge; some papers collect the 2010 to 2021 databases and add most of the feature extraction and classification, which helps to provide better accuracy and the classification result using deep learning and the saturated vector machine algorithm (SVM). The Local Binary Pattern (LBP) and the Principal Component Analysis (PCA) provide good results in the evaluation method [4].

Therefore, the proposed paper reveals the same seven emotions as the facial acting coding system (FACS) through an optimized deep learning algorithm using ECNN. The main goal of the FACS system's development was to identify all potential visible anatomically based face motions. FACS offers a standardised nomenclature for studying face movement, allowing for a wide range of applications. It produces the classification of many facial reactions without employing the optimal technique, such as the seven emotions of the Facial Acting Coding System (FACS). Thus, the proposed system has better accuracy when compared to the existing technique.

The article "Optimal Facial Feature Based Emotional Recognition Using Deep Learning Algorithm" was published in 2022. Journal: Comput Intell Neurosci.

## 2. Objective

The primary goal of this article is to use a deep learning algorithm to recognise different sorts of emotions based on facial features. We do this by implementing seven different types of facial expressions. When compared to the current technique, the feature extraction for our proposed study uses geometric-based approaches, hybrid approaches, holistic approaches, and hybrid approaches, all of which provide improved accuracy.

## 3. Review of the Literature

Yadan Lv et al. [5] in this paper implemented facial recognition via a deep learning algorithm. The parsed components help to detect the various types of the feature recognition technique; therefore, we do not need to add the additional feature for removing noise or any adjusting feature. The parsed technique is one of the most important techniques and a unique technique.

Mehmood et al. [6] in this paper implemented the optimal feature selection and deep learning ensemble methods for emotional recognition from human brain EEG sensors. This paper implements the EEG feature extraction and the feature selection methods based on the optimization of the face recognition technique. Four types of emotional classifications are involved, namely, happy, calm, sad, and scared. The feature extraction is based on the optimal selected feature like the balanced one way ANOVA technique, so it provides better accuracy in the emotional classification. Additional techniques like the arousal-valence space provide enhanced EEG recognition.

Li et al. [7] in this paper implemented the Reliable Crowd-sourcing and deep locality-preserving learning for expression recognition in the wild, for reducing the crowd-sourcing and the new locality loss layer preservation using a deep learning algorithm that is based on the RAFDB face recognition algorithm. Thus, the RAFDB expressed that the five different techniques, such as the calculation of the aged rat and the gender, the second step helps to identify the dimensional space of the image, and the third step helps to identify the two subsets. The first one contains seven types of emotions, and the second subset contains twelve types of emotions. The fourth one is identifying the accuracy, and the fifth one is classifying the images based on the input.

Chen et al. [8] in this paper implemented the Soft-max regression-based deep sparse auto-encoder network for facial emotion recognition in human-robot interaction. This paper implements the SRDSAN technique, which helps to reduce the distortion and identify the learning efficiency and dimensional complexity, whereas the DSAN helps with accurate feature extraction and the soft-max regression helps to classify the input signal.

The article "Optimal Facial Feature Based Emotional Recognition Using Deep Learning Algorithm" was published in 2022. Journal: Comput Intell Neurosci.

Babajee et al. [9] in this paper implemented the identification of human expressions from facial expressions using a deep learning algorithm. This paper proposed the seven types of facial expressions recognition like happy, sad, etc., through deep learning using a convolutional neural network. Thus, this paper contains a dataset of 32,398 for collecting various types of emotional recognition using the Facial Action Coding System (FACS). This paper only depends on the identification method not working as the optimization method.

Hassouneh et al. [10] in this paper implemented the development of a real-time emotional recognition system using facial expressions and EEG based on machine learning and deep neural network methods. This paper implements the optical flow algorithm for identifying facial regression using virtual markers. Therefore, the system of the optical flow algorithm helps to physically challenge people since it recognizes less computational complexity.

Tan et al. [11] in this paper implemented the short-term emotion recognition and understanding based on the spiking neural network modeling of the spatio-temporal EEG patterns using neuro-sense. This paper implements the SNN technique for the very first time. It helps to identify the functions of the brain system. The EEG data are measured by using two techniques like arousal-valence space. The arousal-valence space consists of four types of columns, namely, high arousal, low arousal, and high and low valence space techniques.

Satyanarayana et al. [12] in this paper implemented emotional recognition using deep learning and cloud access. Facial emotional recognition is one of the most important techniques in various applications. The deep learning algorithm plays a vital role in face recognition. Her thesis paper collects various types of emotions like sadness, happiness, calmness, and anger reactions. Therefore, this information goes through the python code, and then it creates its own IP address for every technique.

Jayanthi et al. [13] in this paper implemented an integrated framework for emotional classifications using speech and static images with deep classifier fusion. Emotion recognition is one of the crucial techniques for identifying the stress level in a human being. The two factors that play a crucial role in the identification of the stress level in the human body, namely, emotion recognition and speech modulation.

This paper introduced the integral framework for the calculation of the stress thesis; therefore, this paper includes both emotional recognition and speech modulations in the form of static function, which helps to identify the mental state of human nature. Therefore, this result gives better accuracy when compared to the other algorithms.

The article "Optimal Facial Feature Based Emotional Recognition Using Deep Learning Algorithm" was published in 2022. Journal: Comput Intell Neurosci.

Li et al. [14] in this paper implemented the survey of deep facial expression recognition. Face expression recognition is considered one of the major challenges in the network system. The major challenge in facial expression recognition (FER) is based on the lack of training sets and the unrelatable expression variations. In the very first case, the dataset is arranged in the allocation of the neural pipeline technique. This will help to reduce the challenging issues in the FER technique.

Yadahalli et al. [15] in this paper implemented facial microexpression detection using a deep learning algorithm. This paper collects the eight layers of the dataset while using six types of emotions, namely, happiness, sadness, anger, fear, neutral, and surprised faces. The collected dataset contains the FER model; thus, this paper implies that the FER with a convolutional neural network enhances better accuracy, and the cleared output results in the multimodal facial expression using a single algorithm.

Yang et al. [16] in this paper implemented the three-class emotions recognition based on deep learning using a staked auto-encoder. This paper implements that the EEG signal is measured with discrete entropy calculation methods. The auto-encoder technique in the deep learning algorithm provides better accuracy than the calculation methods in the encoding system. The emotions in this technique are evaluated as the alpha, beta, and gamma values. It gives better accuracy and the classification results by using a deep learning algorithm. Normally, the deep learning algorithm provides good results for the multiple classifications of emotional recognition.

Asaju et al. [17] in this paper implemented the temporal approach to facial emotional expression recognition. This paper implements the various types of emotional recognition in the human body through a deep learning algorithm using a convolutional neural network. The VGG-19 methods are used for feature extraction. Then the facial emotion recognition and the accurate mapping technique are carried out by using the BiL-STM architecture.

Therefore, the CNN- BiL-STM technique is used to evaluate better accuracy and good classification results with the help of the deep learning neural network. Therefore, the Denver Intensity of the Spontaneous Facial Action (DISFA) dataset is used to detect the happy, sad, angry, and neutral faces in the techniques, and then the dataset for the effective state in the E-Environment (DAiSEE) dataset helps to detect the confusion and the irritation.

The article "Optimal Facial Feature Based Emotional Recognition Using Deep Learning Algorithm" was published in 2022. Journal: Comput Intell Neurosci.

Sati et al. [18] in this paper implemented face detection and recognition and face emotion recognition through NVIDIA. Jetson Nano, in this paper implements both face recognition and face emotional detection, traditional to the present facial emotional identifications are one of the most challenging techniques, by adding some features in this technique helps to provide the better accuracy and the classification results. The ANN technique helps to identify and recognize facial emotions.

Rajan et al. [19] in this paper implemented the novel deep learning model for facial expression recognition based on maximum boosted CNN and LSTM and proposed a slightly different model with the boosted FER method, at very first preprocessing methods helps to reduce the noise in the given input function and reduces the dimensionality space function. And then the dual CNN technique is applied, and it becomes more and more boosted. Therefore, this paper finally shows that the combination of the LSTM and MBCNN makes it possible to produce highly accurate feature extraction and classification results.

Mirsamadi et al. [20] in this paper implemented automatic speech emotion recognition using recurrent neural networks. This paper demonstrates that the RNN architecture for feature selection and the novel weighted time pooling strategy are involved in this paper, which helps to increase the salient features extraction.

The IEMOCAP is the new method being used for better classifications in emotional recognition. Therefore, the final results compare the IEMOCAP classifier with the traditional SVM-based SER using fixed design features.

Domnich et al. [21] in this paper implemented the gender bias assessment in emotional recognition based AI method, this paper implements the overview of the facial emotion recognition based on the artificial intelligence method, The SASE- FE dataset is collected based on the gender basis.

Therefore, this dataset is further classified into two types depending on the male and female categories; therefore, each group consists of three neural networks. This process is carried out with the testing and the training phase because some groups are ready to work and some are not available for instant work, and then this work will be split up into three different ways, such as the whole work collection and both female and male data are individually split. Therefore, this function makes us think that the result might be accurate and perfect.

Ekundayo et al. [22] in this paper implemented the multilabel convolution neural network for facial expression recognition and ordinal intensity estimation, as there are many functions that work with the emotional recognition technique such as FER, but none of them is apt for the perfect multiclass emotional classification technique. This paper implements the multilabel convolutional neural network.

The article "Optimal Facial Feature Based Emotional Recognition Using Deep Learning Algorithm" was published in 2022. Journal: Comput Intell Neurosci.

This multiclass emotional classification leads to interclass variation. This problem will be overcome by using enhanced ML-CNN with the Binary Cross Entropy (BEC) loss and the loss from an island. The VGG-16 helps to overcome the fitting process in this technique; therefore, this paper implements the Multilabel Kernel Nearest Neighbor and the MLARAM for feature extraction and the classification is done using a chain classifier.

Wang et al. [23] in this paper implemented the recently advanced technique in deep learning. This paper implements the four-category model for deep learning. The first category consists of deep architectures and convolutional neural networks. The deep neural networks are majorly convinced by the deep learning model. It is one of the most important functions in the machine learning algorithm. It plays a crucial role in the data accuracy and the classification contains both linear and nonlinear specific functions.

The convolutional neural network has three most crucial layers, namely, the convolutional neural layer, the pooling layer, and the fully connected layer. The convolution layer is the very first layer that adds some filters to reduce the noise and the dimensional space in the filter. The pooling layer in the CNN helps to reduce the over-fitting problem. Then the fully connected layer is arranged after the convolutional layer and the pooling layer. Therefore, it removes the inaccurate data in the function.

In this paper Gnana et al. [24] implemented the literature review for the feature selection of high-dimensional data. The simplest way of the feature selection method in the data is set of all data are sent to the statistical measurement approach, therefore this helps to the select the feature selection approach. There are four types of approach involved in the feature selection methods, namely,

1. Wrapped-based methods.
2. Hybrid-based methods.
3. Embedded-based methods.
4. Filter based methods.

## 4. Overview of the Proposed Method

The most widely used method of image analysis is the convolutional neural network (CNN). In contrast to a multilayer perceptron (MLP), CNN has concealed layers known as convolutional layers. The proposed approach is based on the CNN framework with two levels. Background removal, which is utilised to draw out emotions from an image, is the initial stage that is advised. Here, the primary expressional vector is extracted using the standard CNN network module (EV). Finding pertinent facial points of significance leads to the creation of the expressional vector (EV). Changes in expression are closely tied to changes in EV. Using a basic perceptron unit on a facial image with the background removed, the EV is produced. We also include a nonconvolutional perceptron layer as the final level in the FERC model that has been proposed. The input data (or image) is given to each convolutional layer, which modifies it before sending the results to the following layer. A convolutional operation is used in this transformation. It is possible to discover patterns using any of the convolutional layers used. Each convolutional layer contains four filters. Shapes, edges, textures, and objects are typically included in the input image that is supplied to the first-part CNN (used for backdrop removal) in addition to the face. At the beginning of convolutional layer 1, the edge detector, circle detector, and corner detector filters are employed. The second-part CNN filter detects facial features such as the eyes, ears, lips, nose, and cheeks once the face has been identified by using additional filtering methods, such as the median and Gaussian noise filters. As a result, the kernel filter is used in this paper to assist in minimising the borders of the dimensional space. The facial feature is one of the key techniques in emotional recognition, and this paper implements feature extraction using a holistic approach, the hybrid approach, the geometric approach, and the template-based technique. The feature extraction technique is the next stage of the preprocessing technique. As a result, the convolutional neural network receives the output when the feature extraction process is finished. The output continues since the aforementioned feature extraction technique provides the improved CNN model of the facial expression.

The article "Optimal Facial Feature Based Emotional Recognition Using Deep Learning Algorithm" was published in 2022. Journal: Comput Intell Neurosci.

The overview of the proposed method shows that the input image goes through the preprocessing technique. The preprocessing technique helps to reduce the noise in the image.  Figure 1 represents the overview of the proposed ECNN.

### 4.1. Proposed Method

Figure 2 represents the overview of the proposed architecture. The very first dataset contains the various expressions of the facial image; this input goes through the preprocessing technique.

### 4.2. Preprocessing

The kernel filter is one of the most crucial filters in the facial identification of the image; it helps to reduce the unfocus in the image, smooth the edges, and reduce the dimensionality of the image. This work implements the kernel filter for image preprocessing.

One of the most important kernel filter approaches is edge detection, since it predicts the ideal edge and reduces the dimensional space. The smoothening kernel is made up of three different filter evaluations: box, average, Gaussian, and median filters.

The two primary purposes of the preprocessing technique are to

1. add a filter to remove noise and
2. convert an RGB image to a greyscale image.

Edge detection is one of the crucial techniques in the kernel filter since it predicts the perfect edge and reduces the dimensional space. The smoothening kernel consists of the three types of filter evaluation, namely, box, average filter, Gaussian filter, and median filter.

(1) $$\begin{array}{c} \left(f*g\right)\left(a,b\right)=\overset{i=\infty }{\underset{i=-\infty }{\sum }}\overset{\infty }{\underset{j=-\infty }{\sum }}f\left(i,j\right)g\left(a-i,b-j\right)\text{.} \end{array}$$

The edge detection kernels consist of three types of operators, namely, the Prewitt operator, the Sobel operator, and the Laplacian operator. Convolution is the main technique for applying the kernel filter to the input data. Then it measures the error level and applies the needed filter for particular error removal. The smoothening kernel plays an important role in the removal of the noise in the input image.

The Gaussian filter is nothing but a low-pass filter. Normally, the input image suffers from Gaussian noise. This noise will be detected by using the white Gaussian noise filter. The Gaussian noise filter also helps to remove the blurring scale of images. It predicts the accurate image fixation.

(2) $$\begin{array}{c} G\left(u,v\right)=\frac{1}{2*3.14*\phi^{2}}e^{\frac{-\left(u^{2}+v^{2}\right)}{\Psi^{2}}}\text{.} \end{array}$$

(1) shows the Gaussian mathematical expressions in the kernel filter. The median filter is one of the noise-removing filters that helps to reduce noise by adding pepper and salt to the input image.

### 4.3. Feature Extraction

Feature extraction is one of the most crucial techniques in image processing. Therefore, three steps are involved in face recognition, namely, face detection, which is considered as the identification of the input image, followed by face extraction which takes place after the identification of the image. Feature extraction helps to classify the accuracy of the image.

The main function of feature extraction is to reduce the dimensionality of the input images and also reduce the dimensional edges of the image after the completion of feature recognition takes place. Feature recognition is considered the identification of the image. This paper implements the four types of feature recognition [25], namely,

1. Geometric feature-based approach
2. Holistic feature-based approach
3. Hybrid Approach
4. Template-based technique.

#### 4.3.1. Geometric Feature-Based Approach

The size and relative position of the image are involved in working in this process. Normally, geometric-based feature extraction helps to rectify the edge detection and produce a good shape in the image. The canny filter plays a crucial role in this approach. The gradient analysis and the canny filter results are applied to this filter. The canny filter is mainly used for edge detection in the image; the first step for the canny filter is to detect the noise with the Gaussian filter. The gradient magnitude helps smoothen the image after the smoothening threshold process is involved to determine the potential edges. Simply, the geometric feature is defined as the detection of the extracted feature like local features, namely, eyes, eyebrows, nose, and mouth, which are first extracted.

The article "Optimal Facial Feature Based Emotional Recognition Using Deep Learning Algorithm" was published in 2022. Journal: Comput Intell Neurosci.

#### 4.3.2. Holistic Approach

The holistic approach is one of the crucial approaches that detects the whole face in the input, therefore it helps to identify the various emotions in the face, like crying, anger, sadness, happiness, etc. Therefore the application of the holistic approach is wide extended such as Eigen face and the fisher face [26].

#### 4.3.3. Hybrid Approach

The hybrid feature extraction in facial recognition is described as the combination of the hybrid and the all-image feature; it detects accurate facial image recognition, particularly in the form of the eyes, nose, and mouth expressions. This approach involves various techniques in the form of facial expressions, namely,

1. Geometric-based technique
2. Appearance-based technique
3. Template-based technique and the color-based technique.

Figure 3 implies that in the geometric-based approach, the geometric feature technique handles the size and the relative position by using the output of the canny filter and the gradient magnitude.

The appearance-based technique is based on the principal compound analysis (PCA) by using feature extraction. The main function of the PCA is to minimise the huge dimensionality of images into small dimensionality-independent images. It provides the perfect output of the image.

#### 4.3.4. Colour Based Method

The color-based method is mainly focused on red, green, and blue (RGB). The very first step of the preprocessing technique converts the RGB into a greyscale image. Thus, the greyscale image is converted into the binary image by using the valuable threshold values. Therefore, all the processes are completed to remove the color-saturated value calculated. The saturated value is calculated by adding some features to this technique, like the threshold function.

After the completion of the threshold applied in the image, the noise was detected. Then this process handled some open and closed functions such as eyes, ears, and mouth, which were extracted along with some facial functions.

The article "Optimal Facial Feature Based Emotional Recognition Using Deep Learning Algorithm" was published in 2022. Journal: Comput Intell Neurosci.

Figure 4 implements the various types of skin maps from the original image by using the threshold function in the image. This feature extracted image gives the input through the convolutional neural network using the deep learning method.

### 4.4. Convolutional Neural Network

The convolutional neural network is a type of deep learning algorithm. The process of the convolutional neural network is nothing but an integral layer network.

Figure 5 implies that the convolutional neural network performs the multilayer specific task in the form of a classification method. The function of the convolutional neural network is that the input image goes through the RELU layer with convolution and this goes to the maxpooling technique. This process is done again one time, therefore the output image is sent through the fully connected layer. It helps to separate the accurate output. The fully connected layer also helps to classify the image.

The RELU performs the multilayer in a function. Normally, the convolutional layer is used to classify the image. The RELU function in the convolutional neural network helps to separate multiple facial expressions collection. Then it sends the data to the maximum pooling. The maximum pooling helps to reduce the overfitting and the dimensional image and analyze the inaccurate data.

Then the results go through the fully connected layer. This layer is otherwise called the classifying layer.

(3) $$\begin{array}{c} Clarity=\frac{RealPositive}{RealPositive+FakePositive}\text{,}\\ Accuracy=\frac{RP+RN}{RP+RN+FP+FN}\text{.} \end{array}$$

### 4.5. Dataset

The dataset consists of around 32,298 images, each separately labeled. The images are sized in the 48*∗*48 size pixels, thus we used the FER2013 dataset for further analysis. The dataset consists of two-columns, namely, one is a pixel and the other one is emotional [27]. The pixel value is present in the pixel column and the emotional actions are analyzed in the code value from 0–6.

Table 1 shows the dataset for emotions classification using various types of feature extraction.

### 4.6. Testing and Training Model

80% of the data are used as the input of the training phases, therefore the preprocessing technique helps to reduce the noise in the filter. The feature extraction helps to reduce the high dimensionality of the space in the filter. Our paper implements the various types of feature extraction to reduce the dimensional space and the edge detection that are all applied in this paper. Therefore, it produces accurate dimensional quality and clear output images [28]. The classification and the feature extraction work in the same phase in the data. After the classification, the features are transferred from the testing and the training phase [29]. Thus, we collect three models of the training iterations, such as 20, 200, and 600. The training time is 5, 15, and 100.

The article "Optimal Facial Feature Based Emotional Recognition Using Deep Learning Algorithm" was published in 2022. Journal: Comput Intell Neurosci.

Table 2 represents the accuracy rate for the collected data. It shows our proposed method using the CNN technique gives more accurate results when compared to the existing technique [30].

## 5. Results Comparison

The comparison results show that the existing CNN and the SVM technique. The support vector machine-based technique using the Gabor filter, and the Monto Carlo algorithm are used to extract the set of templates [31–45]. The feature extraction of this existing technique does not show perfect results.

Table 3 shows the comparison results for the facial feature recognition; our paper achieves higher accuracy when compared to existing techniques, particularly numerous types of feature extraction, which help to extract the features accurately.

Figure 6 shows the accuracy results for the existing and the proposed method. Thus our proposed method shows better results when compared to the existing technique.

## 6. Conclusion and Future Work

In our study, we proposed the facial feature for emotional recognition using a convolutional neural network through a deep learning algorithm by using different facial features with proper dimensional space reduction, and the edges are sharpened by using the kernel filter in the preprocessing technique. When compared to the current method, the results show improved accuracy and the classification methodology in the convolutional neural network. When comparing our suggested strategy to the current approach, the outcomes are better. It appears that the model's capacity satisfies the challenge of sophisticated facial expression recognition at those resolutions. Using data augmentation techniques such as mixing data from steps (b), (cropping), and (f), as well as adding noise, we can improve the performance of CNN. The featured study entails investigating picture synthesis methods that could be viewed as a deep learning augmentation data solution. It seeks to avoid overfitting for small amounts of data and data hunger. The future of our study hinges on adding more features, identifying ten different types of facial emotions, and researching automatic facial emotion identification.

## Figures and Tables

**Figure 1:** Overview of the proposed ECNN approach.

**Figure 2:** Proposed architecture.

**Figure 3:** Geometric-based approach.

**Figure 4:** Different skin maps in the original image.

The article "Optimal Facial Feature Based Emotional Recognition Using Deep Learning Algorithm" was published in 2022. Journal: Comput Intell Neurosci.

**Figure 5:** Convolutional neural network.

**Figure 6:** Results.

**Table 1:** Emotions tabulations dataset.

Emotions	Code
Happy	0
Sad	1
Surprise	2
Neutral	3
Fear	4
Horror	5
Cry	6

**Table 2:** Accuracy rate.

Epochs	Hrs	Accuracy rate
20	5	80
200	15	95
600	100	97

**Table 3:** Comparison table.

Results	Accuracy rate	Emotions
CNN [30]	79.98	7
SVM [31]	85–90	6
ECNN (proposed method)	97	7

## Data Availability

The datasets used and/or analyzed during the current study are available from the corresponding author upon request.
